# Prognostic Nomograms for Primary High-Grade Glioma Patients in Adult: A Retrospective Study Based on the SEER Database

**DOI:** 10.1155/2020/1346340

**Published:** 2020-07-23

**Authors:** Yi Yang, Mingze Yao, Shengrong Long, Chengran Xu, Lun Li, Yinghui Li, Guangyu Li

**Affiliations:** ^1^Department of Neurosurgery, First Affiliated Hospital of China Medical University, Shenyang 110001, China; ^2^Department of Neurosurgery, Anshan Hospital of the First Hospital of China Medical University, Anshan 114000, China; ^3^Department of Medical Genetics, School of Life Science, China Medical University, Shenyang 110122, China

## Abstract

**Purpose:**

In our study, we aimed to screen the risk factors that affect overall survival (OS) and cancer-specific survival (CSS) in adult glioma patients and to develop and evaluate nomograms.

**Methods:**

Primary high-grade gliomas patients being retrieved from the surveillance, epidemiology and end results (SEER) database, between 2004 and 2015, then they randomly assigned to a training group and a validation group. Univariate and multivariate Cox analysis models were used to choose the variables significantly correlated with the prognosis of high-grade glioma patients. And these variables were used to construct the nomograms. Next, concordance index (C-index), calibration plot and receiver operating characteristics (ROCs) curve were used to evaluate the accuracy of the nomogram model. In addition, the decision curve analysis (DCA) was used to analyze the benefit of nomogram and prognostic indicators commonly used in clinical practice.

**Results:**

A total of 6395 confirmed glioma patients were selected from the SEER database, divided into training set (n =3166) and validation set (n =3229). Age at diagnosis, tumor grade, tumor size, histological type, surgical type, radiotherapy and chemotherapy were screened out by Cox analysis model. For OS nomogram, the C-index of the training set was 0.741 (95% CI: 0.751-0.731), and the validation set was 0.738 (95% CI: 0.748-0.728). For CSS nomogram, the C-index of the training set was 0.739 (95% CI: 0.749-0.729), and the validation set was 0.738 (95% CI: 0.748-0.728). The net benefit and net reduction in inverventions of nomograms in the decision curve analysis (DCA) was higher than histological type.

**Conclusions:**

We developed nomograms to predict 3- and 5-year OS rates and 3- and 5-year CSS rates in adult high-grade glioma patients. Both the training set and the validation set showed good calibration and validation, indicating the clinical applicability of the nomogram and good predictive results.

## 1. Introduction

Among adults, gliomas are the most common primary brain tumors, accounting for more than 70% of primary malignant brain tumors [1–3]. According to the World Health Organization classification criteria, gliomas are categorized as low-grade gliomas (I-II) and high-grade (III-IV) gliomas [4]. The high-grade gliomas are difficult to treat due to their easy invasion of surrounding parenchyma, presenting high mortality and poor prognosis. Many studies explored the factors influencing the prognosis of gliomas, including age at diagnosis, histological type, tumor volume, tumor grade, molecular markers (1p19q-codeletion, IDH state, p53 state, etc.) and the extent of surgical resection. Relevant studies indicated that the survival time of low-grade glioma was long, and the survival time decreased gradually with the increase of tumor grade; besides, the effect of surgical resection on the prognosis was controversial. However, some studies concluded that the extension of surgical resection could effectively improve the prognosis [5–10]. Therefore, based on the above factors, there is no effective method to evaluate the prognosis of primary high-grade gliomas in the course of treatment. There is also a lack of an effective model for predicting the survival of patients with epidemiological data, pathology and surgical treatment.

It is a common statistical method of clinical research to construct the nomogram model of clinical risk factors. The nomogram scores the independent risk factors, then synthesizes into an intuitive scale study model with strong predictability and specificity for the prognosis of the tumor. To date, nomograms have not been applied for adult patients with primary high-grade gliomas.

In summary, we used SEER database to screen multiple independent risk factors, construct nomograms of primary high-grade glioma patients in adult, and perform external validation.

## 2. Methods

### 2.1. Retrieve Information from the SEER Database

All data used in our study came from the SEER database, which has been approved for public use by the local ethics committee. So our study did not require a local ethics approval or a statement. The patients were selected from the SEER database who were diagnosed with primary high-grade glioma from 2004 to 2015 and whose tumor location and histological type codes were referenced in the International Classification of Diseases for Oncology, third edition (ICD-O-3). It was mainly aimed at primary high-grade gliomas in adult, so the inclusion criteria included (1) first primary malignant glioma, eliminating patients with more other primary cancer; (2) age>14; (3) III-IV grades glioma, eliminating unknown classification; (4) major primary sites of gliomas: frontal lobe, temporal lobe, parietal lobe, occipital lobe, overlapping lesion of brain (C71.1, C71.2, C71.3, C71.4, C71.8); (5) major histological types of gliomas: astrocytoma, oligodendroglioma, glioblastoma and mixed glioma (M9400, M9450, M9440, M9382); (6) size of gliomas (it recorded the largest dimension of the primary tumor in millimeters): excluding uncertain records and invalid records, we got a minimun of 1 mm and a maximun of 177 mm; (7) surgical type including no surgery, subtotal resection, gross resection and resection of lobe of brain; (8) laterality including left, right, and not a paired site; (9) excluding patients of unknown race and unknow marital status; (10) specific information on radiotherapy and chemotherapy, eliminating unknown information. A total of 6395 glioma patients were selected according to the screening criteria and randomly divided into a training set of 3166 patients and a validation set of 3229 patients.

The selected variables contained age, gender, race, marital status, tumor grade, site, histological type, tumor size, laterality, surgical type, radiotherapy, chemotherapy, radiation sequence with surgery (Table 1). The OS rates and CSS rates were selected as the research indexes in this study.

### 2.2. Statistics and Analysis of Variables

The optimal cutoff points of age and tumor size were selected by using the X-tile program, and the two continuous variables were converted into classification variables. SPSS 22.0 (IBM) software was used to conduct univariate and multivariate Cox regression model to screen all variables. Statistical significance was accepted at the p <0.05 level. Then seven indicators with significant statistical significance were screened out, including age, tumor grade, histological type, tumor size, surgical type, radiotherapy and chemotherapy (Tables 2 and 3). The Kaplan-Meier method and log-rank test were used for survival analysis. Besides R3.6.1 version was used to draw the survival curves.

### 2.3. Construction and Verification of Nomogram

The nomograms were constructed by the seven indexes screened by statistics. The constructed nomograms were tested by the training set and the validation set, and were evaluated by the C-index, calibration plots and ROC curve, including the degree of differentiation between the predicted value and the true value, the predicted result, as well as the sensitivity and specificity. Moreover, DCA was used to compare the nomograms and histological type, and to test the net benefit and net reduction in inverventions between them. The nomograms and analysis curves were drawn by R3.6.1 version, and the later pictures were combined and arranged by Adobe Illustrator CS6.

## 3. Results

### 3.1. Data from the SEER Database

Table 1 showed the basic information of the selected variables. The median survival time of the training set and the validation set were 10 months and 10 months, and the average survival time were 17.9 and 18.7, the median age were 61 and 61. The X-tile program selected the optimal cutoff points of age and tumor size in the training set. The results of age were 56 years old and 75 years old, and tumor size were 27 mm and 44 mm (Figure 1). In terms of race, whites accounted for more than 90% of the population; the grade of tumor was mainly grade IV, accounting for more than 90%; besides, the primary site of the tumor was mainly frontal lobe, which reached more than 30%; the main histological type was glioblastoma, which reached more than 85%.

### 3.2. Development of the Nomogram

The univariate Cox regression was used to obtain statistically significant indicators including age, marital status, tumor grade, laterality, site, histological type, tumor size, surgical type, radiotherapy, chemotherapy and radiation sequence with surgery, moreover marital status, laterality, site and radiation sequence with surgery were excluded by multivariate Cox regression. Next, the nomograms were constructed based on seven statistically significant indicators: age, tumor grade, size, histological type, surgical type, chemotherapy and radiotherapy (Figure 2). The 3- and 5-year OS rates and 3- and 5-year CSS rates were assessed by nomogram to calculate the corresponding scores. Then, in Table 4, we calculated prognostic risk scores for each risk factor and 3-year, 5-year survival in nomograms (Table 4). According to the OS and CSS scores of each patient in the training set, we used X-tile software to divide the risk scores into three groups, namely low risk, medium risk and high risk (Figure 3).

### 3.3. Effect Verification of Nomogram

We conducted internal evaluation and external validation of the nomograms. The AUC values of the 3- and 5-year OS rates in the training set were 0.767 and 0.778, and in the validation set were 0.759 and 0.768 (Figure 4). The AUC values of the 3- and 5-year CSS rates in the training set were 0.771 and 0.779, and in the validation set were 0.766 and 0.767 (Figure 4). Furthermore, high area under ROC curve was obtained in both groups. The results of the 3- and 5-year OS and CSS rates for both the training set and the validation set in the calibration plots were satisfactory, and the quality of the calibration was high (Figure 5). Moreover, DCA was used to compare the nomograms with the histological type of gliomas, and the net benefit and net reduction in inverventions of nomograms were higher than others in the comparison of 3- and 5-year OS and CSS rates (Figures 6 and 7).

## 4. Discussion

Previous studies have discussed the effect of a single risk factor on the prognosis of gliomas alone, and the number of clinical cases cited was limited, with only single-center, small-sample studies. In our study, from the perspective of multi-center, large-sample, SEER database and nomogram model were combined to predict the 3- and 5-year OS and CSS of primary high-grade glioma patients, and satisfactory results were obtained in external validation. In the verification of nomograms, compared with histological type, the net benefit and net reduction in inverventions of nomograms were higher than the histological type, which further proved the clinical practicability of nomograms. It could be concluded that the constructed nomograms had good value in predicting clinical prognosis.

Our study was based on the epidemiological characteristics of primary high-grade gliomas. First, gliomas were the most common primary intracranial tumor, representing 81% of malignant brain tumors; although relatively rare, they caused significant mortality and poor prognosis [11]. Also, malignant high-grade gliomas were diffusely infiltrative lesions which often infiltrated some important surrounding functional areas and seriously affected the quality of life of patients [12]. However, not all types of gliomas consistently behaved in a malignant fashion, the heterogeneity (in terms of histology, grade, clinical outcomes and genomics) increased the complexity of risk factor research in gliomas [13]. Second, epidemiology had explored a number of potential risk factors, but only genetic factors, ionizing radiation, and a decrease in risk by history of allergies or atopic disease (s) had been shown to be associated with gliomas [2, 14]. Therefore, there are still great defects in the effective prediction of the prognosis of high-grade gliomas.

In the training group, age was statistically significant in the analysis of prognostic factors, with an associated risk of 2.606 (95% CI: 2.288-2.967) for age over 75 years, similar to another study [15]. Moreover, in multivariate cox regression analysis, the differentiation degree of each age group was very significant. Related study has shown that the incidence of gliomas increases with age [16]. It might be related to the decline of the tolerance of the elderly to the operation, because of the poor physical condition of the elderly, the operation would cause great damage to the body. Several studies confirmed that the incidence of cancer increased with age, especially after 65 years [17]. In addition, with the growth of age, the immune system of the elderly would be maladjusted, the function of the anti-tumor system would decline [18], and the repair ability of cells would be weak [19]. These factors led to poor recovery in the elderly after clinical treatment. Race and marital status were more complex factors, such as the encouragement and support from partner [20], different financial circumstances and different comprehensive treatments [21].

Next, in terms of tumor grade, the nomograms included only glioma III and IV, because the prognosis of high-grade gliomas was much worse than that of low-grade gliomas. Compared with low-grade gliomas, the high-grade gliomas exhibited a high degree of vigorous growth and tumor angiogenesis increased. [22] This might be related to III/IV glioma patients with high expression of O6-methylguanine-DNA-methyltransferase (MGMT) promoter methylation, 1p19q co-deletion, isocitrate dehydrogenase (IDH) gene mutations [23]. Likewise, gain of 19p and grade III histology were negatively correlated with the prognosis of patients with gliomas [24].

Then, for histological type, the multivariate cox regression analysis showed that the prognosis of glioblastomas and astrocytomas were worse than other types. Glioblastomas had a high degree of malignancy and were characterized by rapid proliferation and strong invasiveness [25]. High expresssion of CD44 [26] and lower expression level of CNTN3 [27] were both related to the poor prognosis of glioblastomas. Besides, astrocytomas might be related to the fact that TN-C immunopositivity was noted in the ECM of the fibrotic stroma in highly malignant brain tumors and along the tumor border especially in high-grade astrocytomas [28] or PDok2 protein was highly expressed [29].

In our study, the site of high-grade gliomas was only statistically significant in univariate cox regression analysis. The frontal lobe was the major primary site of gliomas, which might be related to the gene expression of the gliomas [30]. Relevant study had shown that when most glioma patients tested positive for FFT-1, the tumor was mostly involved in the frontal lobe [31]. Also the primary site of the tumor was associated with the surgical type, for example, the brain stem, which had a high postoperative mortality rate, had very limited surgical options [32].

Also in terms of tumor size, the associated risk increased with the increase of tumor size, because much other factors were considered for this risk factor [33]. For example, the larger glioma could only be treated with chemoradiotherapy or partial resection due to the wide range of infiltration and more invasion of surrounding parenchymal areas. In contrast, the treatment of small gliomas was more selective, and the extensive resection could be used for reference. However, this kind of operation had a great damage to patients and also affected the survival time of patients, the tumor size as a risk factor needed further study.

Among the relevant risk factors studied, the influence of surgical resection range on prognosis was controversial. [34] It was well known that extent of resection affected clinical outcomes together with OS [35]. The surgical types of brain tumors were selected for analysis. According to the survival analysis curve (Figure 8), gross resection was significantly differentiated from subtotal resection, and resection of lobe of brain and gross resection had similar effects. However, clinical evidences for surgical types selection were lacking, and evidences supporting the use of extended resection of gliomas were still insufficient, particularly in lower-grade gliomas where neurological deficits could result in long-term disability [36]. However, some studies still suggested that more extensive resection of both low-grade and high-grade gliomas could improve OS, progression-free survival and superior quality of life [32, 37–40]. Survival time, functional recovery and tumor recurrence rate all improved with the increase of resection range [3, 41]. Some studies have sought to identify predictors of postoperative seizure control after surgical resection of gliomas; gross-total resection was shown to be a significant predictor in this respect [42–45]. Significant resection of diffuse, infiltrating low-grade gliomas maximized seizure control and did not necessarily cause permanent neurological deficits [46]. In addition, gross resecction has been found to be effective in the control of postoperative epilepsy [47, 48]. In general, the risk factor of surgical type remained to be studied, and resection of lobe of brain was also collected in SEER database and found to be statistically significant, making it a promising research direction.

In this study, radiotherapy and chemotherapy were also important prognostic factors. In clinical practice, radiotherapy was generally used for 2 to 3 cm invasive tumors. In a clinical trial of glioblastoma, the median survival time for patients receiving radiotherapy alone was 12.1 months, similar to the median survival time in this study [49]. In addition, patients with MGMT methylated had better progression-free and overall survival than those without methylation when treated with radiotherapy and temozolomide [50]. Another study of oligodendrogliomas showed significant improvenments in survival in patients receiving chemotherapy with procarbazine, vincristine and lomustine [51, 52]. Moreover, we compared the effects of surgery and radiation therapy on prognosis (Figure 9). It was clear that a combination of surgery and chemotherapy has the best prognosis. Interestingly, chemotherapy is better than surgery in the long run. This might be related to the older age of the patients, the greater degree of malignancy of the tumor and the greater harm of the operation to the patinets. Therefore, in clinical practice, for patients with high-grade gliomas, the conservative treatment such as chemotherapy should be adopted, and the choice of surgery needs to be cautious.

Nonetheless, our study has some shortcomings. Due to the incomplete genetic records of patients in the SEER database, there was a lack of gene-level studies. Also, SEER did not provide detailed information on postoperative radiotherapy and chemotherapy, whether there was recurrence or not, which might lead to certain limitations of the study results. More importantly, the SEER database did not provide the scope or volume of surgical resection. In terms of racial selection, whites were the majority. Inevitably there was racial heterogeneity. Only representative sites and partial histologic types of gliomas were selected, so some special sites and rare histologic types of gliomas were not discussed.

## 5. Conclusions

Based on the SEER database, our study used several independent risk factors to establish nomograms of 3- and 5-year OS and CSS rates for primary high-grade glioma patients and external validations were performed to ensure the accuracy and reliability of the constructed nomograms. Nomograms could estimate survival precisely and provide risk assessments for further treatment of patients with primary high-grade gliomas.

## Figures and Tables

**Figure 1:** The results of the X-tile program for optimal cutoff points of age and tumor size. X-tile plot of all patients is displayed in the figure, the age optimal cutoff value marked by the black circle in the (a) is shown by a histogram of the entire cohort (c), and a Kaplan–Meier plot (e); the size optimal cutoff value marked by the black circle in the (b) is shown by a histogram of the entire cohort (d), and a Kaplan–Meier plot (f). The figure shows the optimal cutoff points for adult patients with gliomas (56 and 75; 27 and 44 mm).

**Figure 2:** The nomograms of the prediction of 3- and 5-year OS and CSS in adult glioma patients based on the training set.

**Figure 3:** The results of the X-tile program for optimal cutoff points of risk scores. X-tile plot of all patients is displayed in the figure, the risk scores optimal cutoff value of OS marked by the black circle in the (a) is shown by a histogram of the entire cohort (c), and a Kaplan–Meier plot (e); the risk scores optimal cutoff value of CSS marked by the black circle in the (b) is shown by a histogram of the entire cohort (d), and a Kaplan–Meier plot (f). The figure shows the optimal cutoff points for risk scores (87 and 123; 82 and 116).

**Figure 4:** Calibration plots of the nomogram for 3- and 5-year OS (a, b) prediction in the training set, 3- and 5-year OS (c, d) prediction in the validation set, 3- and 5-year CSS (e, f) prediction in the training set and 3- and 5-year CSS (g, h) prediction in the validation set.

**Figure 5:** Discriminatory accuracy for predicting OS assessed by receiver operator characteristics (ROC) analysis calculating area under the curve (AUC). The 3- and 5-year OS in the training set (a, b) and 3- and 5-year OS in the validation set (c, d). The 3- and 5-year CSS in the training set (e, f) and 3- and 5-year CSS in the validation set (g, h).

**Figure 6:** Decision curve analysis for the nomograms and histologic type of training set. Figure (a) and (c) are the new benefit curves of 3- and 5-year OS rates of training set. Figures (b) and (d) are the net reduction for intervention curves of the 3- and 5-year OS rates of the training set. Figure (e) and (g) are the new benefit curves of 3- and 5-year CSS rates of training set. Figures (f) and (h) are the net reduction for intervention curves of the 3- and 5-year CSS rates of the training set.

**Figure 7:** Decision curve analysis for the nomograms and histologic type of validation set. Figure (a) and (c) are the new benefit curves of 3- and 5-year OS rates of validation set. Figures (b) and (d) are the net reduction for intervention curves of the 3- and 5-year OS rates of the validation set. Figure (e) and (g) are the new benefit curves of 3- and 5-year CSS rates of validation set. Figures (f) and (h) are the net reduction for intervention curves of the 3- and 5-year CSS rates of the validation set.

**Figure 8:** Survival analysis curve for surgical types of the nomograms of training and validation set. Figure (a) is the survival analysis curve of OS in training set. Figure (b) is the survival analysis curve of OS in validation set. Figure (c) is the survival analysis curve of CSS in training set. Figure (d) is the survival analysis curve of CSS in validation set.

**Figure 9:** Survival analysis curve for surgery and chemotherapy of the nomograms of training and validation set. Figure (a) is the survival analysis curve of OS in training set. Figure (b) is the survival analysis curve of OS in validation set. Figure (c) is the survival analysis curve of CSS in training set. Figure (d) is the survival analysis curve of CSS in validation set.

**Table 1:** Baseline characteristics of glioma patients from SEER database.

Patient characteristics	All patients	Training set	Validation set
	N =6395	N =3166	N =3229
	No. of patients(%)	No. of patients(%)	No. of patients(%)
Age(years)			
<56	2328 (36.4)	1156 (36.5)	1172 (36.3)
56-75	3115 (48.7)	1543 (48.7)	1572 (48.7)
>75	952 (14.9)	467 (14.8)	485 (15.0)
Gender			
Male	3754 (58.7)	1850 (58.4)	1904 (59.0)
Female	2641 (41.3)	1316 (41.6)	1325 (41.0)
Race			
White	5788 (90.5)	2882 (91.0)	2906 (90.0)
Black	320 (5.0)	153 (4.8)	167 (5.2)
Other^a^	287 (4.5)	131 (4.1)	156 (4.8)
Marital status			
Married	4204 (65.7)	2099 (66.3)	2105 (65.2)
Single	945 (14.8)	464 (14.7)	481 (14.9)
Separated/Divorced	633 (9.9)	296 (9.3)	337 (10.4)
Widowed	613 (9.6)	307 (9.7)	306 (9.5)
Grade			
GradeIII	603 (9.4)	292 (9.2)	311 (9.6)
GradeIV	5792 (90.6)	2874 (90.8)	2918 (90.4)
Laterality			
Left	2798 (43.8)	1388 (43.8)	1410 (43.7)
Right	2861 (44.7)	1425 (45.0)	1436 (44.5)
Not a paired site	736 (11.5)	353 (11.1)	383 (11.9)
Site			
C71.1Frontal lobe	2100 (32.8)	1050 (33.2)	1050 (32.5)
C71.2Temporal lobe	1719 (26.9)	838 (26.5)	881 (26.3)
C71.3Parietal lobe	1194 (18.7)	596 (18.8)	598 (18.5)
C71.4Occipital lobe	280 (4.4)	139 (4.4)	141 (4.4)
C71.8Overlapping lesion	1102 (17.2)	543 (17.2)	559 (17.3)
Histological			
Mixed glioma	368 (5.8)	174 (5.5)	194 (6.0)
Astrocytoma	321 (5.0)	171 (5.4)	150 (4.6)
Glioblastoma	5622 (87.9)	2788 (88.1)	2834 (87.8)
Oligodendroglioma	84 (1.3)	33 (1.0)	51 (1.6)
Size(mm)			
<26	855 (13.4)	439 (13.9)	416 (12.9)
27-44	2144 (33.5)	1045 (33.0)	1099 (34.0)
>44	3396 (53.1)	1682 (53.1)	1714 (53.1)
Surgery			
No surgery	1123 (17.6)	580 (18.3)	543 (16.8)
Subtotal resection	1875 (29.3)	930 (29.4)	945 (29.3)
Gross resection	993 (15.5)	496 (15.7)	497 (15.4)
Resection of lobe of brain	2404 (37.6)	1160 (36.6)	1244 (38.5)
Radiotherapy			
Yes	4897 (76.6)	2422 (76.5)	2475 (76.6)
No/unknown	1498 (23.4)	744 (23.5)	754 (23.4)
Chemotherapy			
Yes	4402 (68.8)	2172 (68.6)	2230 (69.1)
No/unknown	1993 (31.2)	994 (31.4)	999 (30.9)
Radiation sequence with surgery			
Prior to surgery	22 (0.3)	13 (0.4)	9 (0.3)
After surgery	4171 (65.2)	2042 (64.5)	2129 (65.9)
Before and after	28 (0.4)	12 (0.4)	16 (0.5)
Unknown	2174 (34.0)	1099 (34.7)	1075 (33.3)

^a^Including American Indian/Alaskan native and Asian/Pacific islander.

**Table 2:** Univariate and multivariate Cox regression analysis of factors associated with OS in the training set (n =3166).

Variable	Univariate analysis			Multivariate analysis		
	*P value*	HR	95% CI	*P value*	HR	95% CI
Age(years)	<0.001	2.003	1.892-2.121	<0.001		
<56				Reference		
56-75				<0.001	1.755	1.607-1.915
>75				<0.001	2.606	2.288-2.967
Gender	0.638	1.018	0.945-1.098			
Male						
Female						
Race	0.189	0.945	0.869-1.028			
White						
Black						
Other						
Marital status	<0.001	1.140	1.098-1.185	0.095		
Married				Reference		
Single				0.278	1.064	0.951-1.191
Separated/Divorced				0.581	1.038	0.910-1.184
Widowed				0.017	1.171	1.029-1.333
Grade	<0.001	1.575	1.375-1.805			
GradeIII				Reference		
GradeIV				<0.001	1.306	1.131-1.508
Laterality	0.001	1.099	1.038-1.164	0.247		
Left				Reference		
Right				0.604	0.979	0.904-1.061
Not a paired site				0.145	1.153	0.952-1.395
Site	<0.001	1.088	1.060-1.117	0.248		
C71.1Frontal lobe				Reference		
C71.2Temporal lobe				0.150	0.930	0.843-1.027
C71.3Parietal lobe				0.127	0.919	0.825-1.024
C71.4Occipital lobe				0.429	1.080	0.893-1.306
C71.8Overlapping lesion				0.804	1.021	0.865-1.207
Histological	<0.001	1.521	1.418-1.632	<0.001		
Mixed glioma				Reference		
Astrocytoma				<0.001	3.242	2.469-4.257
Glioblastoma				<0.001	4.707	3.747-5.914
Oligodendroglioma				0.102	0.621	0.351-1.100
Size(mm)	0.001	1.088	1.033-1.145	<0.001		
<26				Reference		
27-44				0.033	1.141	1.011-1.287
>44				<0.001	1.344	1.198-1.508
Surgery	<0.001	0.817	0.790-0.846	<0.001		
No surgery				Reference		
Subtotal resection				<0.001	0.584	0.491-0.694
Gross resection				<0.001	0.444	0.367-0.538
Resection of lobe of brain				<0.001	0.564	0.476-0.670
Radiotherapy	<0.001	2.164	1.984-2.360			
Yes				Reference		
No/unknown				<0.001	1.578	1.305-1.909
Chemotherapy	<0.001	2.163	1.997-2.343			
Yes				Reference		
No/unknown				<0.001	1.688	1.514-1.881
Radiation sequence with surgery	<0.001	1.495	1.438-1.554	0.736		
Prior to surgery				Reference		
After surgery				0.459	0.813	0.470-1.407
Before and after				0.510	0.757	0.330-1.734
Unknown				0.677	0.884	0.495-1.578

Abbreviations: OS: overall survival; CSS: cancer-specific survival; HR: hazard ratio; CI: confidence interval.

**Table 3:** Univariate and multivariate Cox regression analysis of factors associated with CSS in the training set (n =3166).

Variable	Univariate analysis			Multivariate analysis		
	*P value*	HR	95% CI	*P value*	HR	95% CI
Age(years)	<0.001	1.968	1.856-2.087	<0.001		
<56				Reference		
56-75				<0.001	1.696	1.551-1.856
>75				<0.001	2.509	2.195-2.869
Gender	0.370	1.036	0.959-1.119			
Male						
Female						
Race	0.176	0.942	0.863-1.027			
White						
Black						
Other						
Marital status	<0.001	1.132	1.089-1.178	0.140		
Married				Reference		
Single				0.431	1.048	0.933-1.177
Separated/divorced				0.845	1.014	0.885-1.162
Widowed				0.023	1.169	1.022-1.337
Grade	<0.001	1.604	1.393-1.847			
GradeIII				Reference		
GradeIV				0.001	1.301	1.121-1.509
Laterality	0.013	1.078	1.016-1.143	0.371		
Left				Reference		
Right				0.388	0.964	0.888-1.047
Not a paired site				0.357	1.097	0.901-1.335
Site	<0.001	1.085	1.057-1.114	0.108		
C71.1Frontal lobe				Reference		
C71.2Temporal lobe				0.078	0.913	0.825-1.010
C71.3Parietal lobe				0.099	0.911	0.815-1.018
C71.4Occipital lobe				0.309	1.105	0.911-1.340
C71.8Overlapping lesion				0.752	1.028	0.867-1.219
Histological	<0.001	1.553	1.444-1.671	<0.001		
Mixed glioma				Reference		
Astrocytoma				<0.001	3.198	2.399-4.262
Glioblastoma				<0.001	5.018	3.951-6.374
Oligodendroglioma				0.100	0.599	0.325-1.104
Size(mm)	0.003	1.085	1.029-1.143	<0.001		
<26				Reference		
27-44				0.047	1.134	1.002-1.283
>44				<0.001	1.339	1.190-1.507
Surgery	<0.001	0.817	0.789-0.847	<0.001		
No surgery				Reference		
Subtotal resection				<0.001	0.576	0.481-0.690
Gross resection				<0.001	0.439	0.360-0.534
Resection of lobe of brain				<0.001	0.556	0.466-0.665
Radiotherapy	<0.001	2.126	1.943-2.326			
Yes				Reference		
No/unknown				<0.001	1.571	1.290-1.913
Chemotherapy	<0.001	2.141	1.972-2.325			
Yes				Reference		
No/unknown				<0.001	1.704	1.524-1.906
Radiation sequence with surgery	<0.001	1.487	1.428-1.547	0.727		
Prior to surgery				Reference		
After surgery				0.376	0.781	0.451-1.351
Before and after				0.508	0.755	0.330-1.732
Unknown				0.566	0.843	0.471-1.509

Abbreviations: OS: overall survival; CSS: cancer-specific survival; HR: hazard ratio; CI: confidence interval.

**Table 4:** Prognostic risk score from nomograms.

Variable	Risk score of OS	Risk score of CSS
Age(years)		
<56	0	0
56-75	28	25
>75	50	46
Grade		
GradeIII	0	0
GradeIV	14	13
Histological		
Mixed glioma	23	23
Astrocytoma	82	79
Glioblastoma	100	100
Oligodendroglioma	0	0
Size(mm)		
<26	0	0
27-44	8	7
>44	17	16
Surgery		
No surgery	46	45
Subtotal resection	45	14
Gross resection	0	0
Resection of lobe of brain	13	12
Radiotherapy		
Yes	0	0
No/unknown	26	24
Chemotherapy		
Yes	0	0
No/unknown	28	27
3-year survival probability		
0.9	15	18
0.5	106	106
0.1	165	162
5-year survival probability		
0.9	2	6
0.5	93	94
0.1	152	150

Abbreviations: OS: overall survival; CSS: cancer-specific survival.

## Data Availability

In our study, all data were selected from the Surveillance, Epidemiology, and End Results (SEER) database at https://seer.cancer.gov/. Relevantdata can be accessed through proper request, from the first author.

## Abbreviations

OS: Overall survival
CSS: Cancer-specific survival
HR: Hazards ratio
CI: Confidence interval
ROC: Receiver-operating characteristic
AUC: Area under the curve
C-index: Concordance index
DCA: Decision curve analysis
SEER: Surveillance, epidemiology, and end results.
